# DCNN-FuzzyWOA: Artificial Intelligence Solution for Automatic Detection of COVID-19 Using X-Ray Images

**DOI:** 10.1155/2022/5677961

**Published:** 2022-08-09

**Authors:** Abbas Saffari, Mohammad Khishe, Mokhtar Mohammadi, Adil Hussein Mohammed, Shima Rashidi

**Affiliations:** ^1^Department of Electrical Engineering, Imam Khomeini Marine Science University, Nowshahr, Iran; ^2^Department of Information Technology, College of Engineering and Computer Science, Lebanese French University, Erbil, Kurdistan Region, Iraq; ^3^Department of Communication and Computer Engineering, Faculty of Engineering, Cihan University-Erbil, Erbil, Kurdistan Region, Iraq; ^4^Department of Computer Science, College of Science and Technology, University of Human Development, Sulaymaniyah, Kurdistan Region, Iraq

## Abstract

Artificial intelligence (AI) techniques have been considered effective technologies in diagnosing and breaking the transmission chain of COVID-19 disease. Recent research uses the deep convolution neural network (DCNN) as the discoverer or classifier of COVID-19 X-ray images. The most challenging part of neural networks is the subject of their training. Descent-based (GDB) algorithms have long been used to train fullymconnected layer (FCL) at DCNN. Despite the ability of GDBs to run and converge quickly in some applications, their disadvantage is the manual adjustment of many parameters. Therefore, it is not easy to parallelize them with graphics processing units (GPUs). Therefore, in this paper, the whale optimization algorithm (WOA) evolved by a fuzzy system called FuzzyWOA is proposed for DCNN training. With accurate and appropriate tuning of WOA's control parameters, the fuzzy system defines the boundary between the exploration and extraction phases in the search space. It causes the development and upgrade of WOA. To evaluate the performance and capability of the proposed DCNN-FuzzyWOA model, a publicly available database called COVID-Xray-5k is used. DCNN-PSO, DCNN-GA, and LeNet-5 benchmark models are used for fair comparisons. Comparative parameters include accuracy, processing time, standard deviation (STD), curves of ROC and precision-recall, and F1-Score. The results showed that the FuzzyWOA training algorithm with 20 epochs was able to achieve 100% accuracy, at a processing time of 880.44 s with an F1-Score equal to 100%. Structurally, the i-6c-2s-12c-2s model achieved better results than the i-8c-2s-16c-2s model. However, the results of using FuzzyWOA for both models have been very encouraging compared to particle swarm optimization, genetic algorithm, and LeNet-5 methods.

## 1. Introduction

COVID-19 was initially designated an epidemic disease by the World Health Organization (WHO) in March 2020 [1]. Due to the increasing number of deaths, the spread of the disease, the lack of access to vaccines and particular drugs, and rapid diagnosis of the disease to break, the transmission chain has become one of the most important research topics for researchers. Polymerase chain reaction (PCR) test [2] and X-ray images [3] are standard methods in detecting COVID-19. One of the problems of PCR tests is that there are not enough kits and also it takes a relatively long time to answer the test. In addition to being affordable, X-ray images are always and everywhere available. Reducing the time to diagnose and detect positive cases, even without fever and cough symptoms, are other benefits of using X-ray images [4]. AI tools can increase processing time and high accuracy in detecting patients with COVID-19 [5]. Much research has been done to identify positive cases of COVID-19 [3, 6]. However, until COVID-19 disease is completely eradicated, the need to research and discover new, fast, low-cost, and accurate techniques is acute. DL is one of the AI techniques for detecting positive cases of COVID-19 [7]. Training is the most challenging part of DL. Examples of algorithms used for DL training are conjugate gradient (CG) algorithm [8], Krylov subspace descent (KSD) algorithm [9], and Hessian-free optimization (HFO) approach [10].

While stochastic GDB training methods are simple to construct and run quickly in the producer for large numbers of training samples, GDB approaches require extensive manual parameter adjustment for optimal performance. Their structure is sequential and leads to parallelizing them with GPU become challenging. On the other hand, though CG methods are stable for training, they are almost slow lead to needing multiple CPUs and a lot of RAMs resource [8]. Deep auto-encoders used HFO to train the weights of standard CNNs, which performs better than Hinton and Salakhutdinov's approach for pretraining and fine-tuning deep auto-encoders [11]. In addition, HFO is weaker than KSD and more complex. In terms of the amount of memory required, HFO requires less memory than KSD. KSD optimization and classification speeds also work better [9]. Recent years have seen the employment of metaheuristic and evolutionary algorithms to solve and optimize real-world problems [12–14]. Despite this, research on optimizing DL training needs to be given more attention. Optimization based on metaheuristic algorithms with a hybrid genetic algorithm and DCNN is the beginning of this field study [15]. This model determines the DCNN parameters through GA's crossover and mutation processes, with the DCNN structure modeled as a chromosome in GA. Alternatively, only the weights and biases of the first convolution layer (*C*1) and the third convolution layer (*C*3) are used as chromosomes during the crossover step. In [16], they present an evolutionary method for fine-tuning the parameters of a DCNN by utilizing the Harmony Search (HS) algorithm and several of its improved variants for handwritten field digit and fingerprint detection. In [17], researchers will develop a hybrid deep neural network (DNN), using computed tomography (CT) and X-ray imaging, to predict the risk of COVID-19-related disease onset. In [18], a new method of diagnosing COVID-19 based on chest X-ray images using artificial intelligence is proposed. In comparison to the state-of-the-art techniques currently used, the proposed method will demonstrate outstanding performance.

In [19], the progressive unsupervised learning (PAUL) algorithm is used for DCNN training. PUL is the easiest way to implement. Therefore, it is considered a primary benchmark for unsupervised feature learning. Due to the fact that clustering data sets might be difficult to categorize, PUL initially inserts a selection stage between the clustering and fine-tuning stages. In [20], an approach for automatically building DCNN architectures on the basis of GA is suggested for optimizing image classification. The lack of knowledge about the structure of DCNN is the most crucial feature of this method. In contrast, the presence of large DCNNs causes chromosomes to grow, thus slowing down the algorithm. Due to the faults described, our proposed strategy comprises training a DCNN model on Data 1 to identify positive and negative cases of COVID-19 samples using X-ray pictures. Following that, the previously trained DCNN's FCL will be replaced with the new FCL, which has been tuning using the whale optimization algorithm, and employs fuzzy logic to adjust its control parameters for better WOA development and performance. The name of the proposed algorithm is called FuzzyWOA. Therefore, in this article, our main motivation is to investigate the impact of FuzzyWOA on improving DCNN performance. Our main contribution in this paper is to improve WOA performance by designing and applying a fuzzy system to balance the exploration and extraction boundaries in the search space for automatic detection of COVID-19 using X-ray images. In this regard, for a fairer comparison, in addition to FuzzyWOA, PSO, GA, and LeNet-5 are used for two DCNN models with different structures in order to automatically detect COVID-19 cases. Of course, it should be noted that various metaheuristic methods have been used to train the neural network, such as sine-cosine algorithm [21], Salp swarm algorithm [22], best-mass gravitational search algorithm [23], particle swarm optimizer [24], biogeography-based optimization [25], dragonfly algorithm [26], and chimp optimization algorithm [27]. But the common problem of these algorithms that leads to inefficiency in some problems is the lack of detection of two phases of exploration and extraction. One of the advantages of using FuzzyWOA is establishing a correct trade-off between the two phases of exploration and extraction in the algorithm's search space. Other disadvantages of using some high metaheuristic methods include being stuck in local optimizations, low convergence speed, high complexity, increasing the number of control parameters, and so on. For this reason, it seems necessary to use an algorithm that performs better in less time. Improvements to FuzzyWOA have eliminated all of these drawbacks. Following that, the other connection weights are kept in the residual layers of the pretrained DCNN, resulting in the training of a linear structure using the characteristics of the final layer.

## 2. Materials and Methods

This section consists of four subsections. The first subsection first introduces WOA and then describes the proposed FuzzyWOA algorithm. The second subsection deals with the DCCN model. The third subsection is about the COVID X-ray database, and the fourth subsection describes the methodology.

### 2.1. FuzzyWOA

First, the WOA mathematical model is explained, and then how to use fuzzy logic to develop the algorithm.

#### 2.1.1. WOA

The WOA optimization algorithm was introduced in 2016, inspired by the way whales were hunted by Mirjalili and Lewis [28]. WOA begins with a collection of randomly generated solutions. Each iteration, the search agents update their location by using three operators: encircling prey, bubble-net assault (extraction phase), and bait search (exploration phase). Whales discover and encircle prey. The WOA assumes that the best solution right now his prey. That once best search agent has been recognized, all other search agents' locations will be updated to point to the best search agent. This behavior is expressed by the following equations:

(1) $$\begin{array}{c} \overset{⟶}{D}=\left|\overset{⟶}{C}.\overset{⟶}{X^{*}}\left(t\right)-\overset{⟶}{X}\left(t\right)\right|, \end{array}$$

(2) $$\begin{array}{c} \overset{⟶}{X}\left(t+1\right)=\overset{⟶}{X^{*}}\left(t\right)-\overset{⟶}{A}.\overset{⟶}{D}, \end{array}$$

where *t* is the current iteration, $\overset{⟶}{A}$ and $\overset{⟶}{C}$ are the coefficient vectors, ($\overset{⟶}{X^{*}}$) is the place vector is the best solution so far, and $\overset{⟶}{X}$ is the place vector. In each iteration of the algorithm, ($\overset{⟶}{X^{*}}$) should be updated if a better answer is reached. The vectors $\overset{⟶}{A}$ and $\overset{⟶}{C}$ are obtained using the following equations:

(3) $$\begin{array}{c} \overset{⟶}{A}=2\overset{⟶}{\alpha }.\overset{⟶}{r}-\overset{⟶}{\alpha }, \end{array}$$

(4) $$\begin{array}{c} \overset{⟶}{C}=2.\overset{⟶}{r}, \end{array}$$

where $\overset{⟶}{\alpha }$ decreases linearly from 2 to zero during repetitions and $\overset{⟶}{r}$ is a random vector in the distance [0, 1]. The whale uses the bubble-net assault strategy to swim simultaneously around its target and along a contraction circle in a spiral pattern. To describe this concurrent behavior, it is anticipated that the whale would change its location during optimization via one of the contractile siege mechanisms or the spiral model with a 50% probability. Equation (5) defines the mathematical model for this phase.

(5) $$\begin{array}{c} \overset{⟶}{X}\left(t+1\right)=\left\{\begin{array}{c} \overset{⟶}{X^{*}}\left(t\right)-\overset{⟶}{A}.\overset{⟶}{D}\text{if}p<0.5\\ \overset{⟶}{D}.e^{bi}.\;\cos\left(2\pi l\right)\text{if }p\geq 0.5 \end{array},\right. \end{array}$$

where $\overset{⟶}{D}\;$ is obtained from equation (6) and refers to the distance *i* from the whale to the prey (the best solution ever obtained). A constant *b* is used to specify the geometry of the logarithmic helix, and *l* is a random value between −1 and 1. p is a nonzero integer between 0 and 1. Vector *A* is used with random values between −1 and 1 to bring search agents closer to the reference whale. In the search for prey to update the search agent's position, random agent selection is used instead of using the best search agent's data. The mathematical model is in the form of the following equations:

(6) $$\begin{array}{c} \overset{⟶}{D}=\left|\overset{⟶}{C}\right|.\overset{⟶}{X_{ran\;d}}.\overset{⟶}{X}, \end{array}$$

(7) $$\begin{array}{c} \overset{⟶}{X}\left(t+1\right)=\overset{⟶}{X_{ran\;d}}-\overset{⟶}{A}.\overset{⟶}{D}, \end{array}$$

$\overset{⟶}{X_{ran\;d}}$ is the randomly chosen position vector (random whale) for the current population, and vector $\overset{⟶}{A}$ is utilized with random values larger or equal to one to drive the search agent away from the reference whale [29].

#### 2.1.2. Proposed Fuzzy Logic for Tuning Control Parameters

The proposed fuzzy model receives the normalized performance of each whale in the population (normalized fitness value) and the current values of the parameters $\overset{⟶}{\alpha }$ and $\overset{⟶}{C}$. The output also shows the amount of change using the symbols Δ*α* and Δ*C*. The NFV value for each whale is obtained by equation (8).

(8) $$\begin{array}{c} \text{NFV}=\frac{\text{fitness}-{\text{fitness}}_{\min}}{{\text{fitness}}_{\min}-{\text{fitness}}_{\max}}. \end{array}$$

The NFV value is in the range of [0.1]. This paper's optimization problem is of the minimization type, in which the fitness of each whale is obtained directly by the optimal amount of these functions. Equations (9) updating the parameters $\overset{⟶}{\alpha }$ and $\overset{⟶}{C}$ for each whale are as follows:

(9) $$\begin{array}{c} {\overset{⟶}{\alpha }}^{t+1}={\overset{⟶}{\alpha }}^{t}+\Delta \alpha \\ {\overset{⟶}{C}}^{t+1}={\overset{⟶}{C}}^{t}+\Delta C. \end{array}$$

The fuzzy system is responsible for updating the parameters $\overset{⟶}{\alpha }$ and $\overset{⟶}{C}$ of each member of the population (whale), and the three inputs of this system are the current value of parameters $\overset{⟶}{\alpha }$, $\overset{⟶}{C}$, and NFV. Initially, these values are “fuzzification” by membership functions. Then their membership value is obtained using *μ*. These values are applicable to a set of rules and result in the values ∆*α* and ∆*C*. Following the determination of these values, the “defuzzification” technique is used to approximate the numerical values ∆*α* and ∆C. Finally, these values are applied in equations (9) and (10) to update the parameters ∆*α* and ∆*C*. The fuzzy system used in this article is of the Mamdani type (see Table 1). The suggested fuzzy model and membership functions used to update the whale algorithm's control parameters are shown in Figure 1.

### 2.2. Convolutional Neural Network

DCNNs are very similar to multilayer perceptron neural networks [30]. These networks are built on the basis of three principles: weight sharing between connections, local receive fields, and temporal/spatial subsampling [31, 32]. The principles discussed above may be classified into two types of layers: subsampling layers and convolution layers. Three convolution layers *C*1, *C*3, and *C*5, positioned between layers *S*2 and *S*4, and a final output layer *F*6 comprise the processing layers (as shown in Figure 2). Feature maps are used to arrange these subsampling and convolution layers. In the last layer, neurons in the convolution layer are connected to a local receptive field. Thus, neurons with the same feature maps (FMs) receive data from different input regions until the input is wholly skimmed to share identical weights. The FMs are spatially downsampled by a factor of two in the subsampling layer. For example, in subsequent layer *S*4, FM of size 10 × 10 is subsampled to conforming FM of size 5 × 5. The last layer is responsible for categorization (*F*6). Each FM in this structure is the result of convolution between the maps of the previous layer and their respective kernel and a linear filter. The weights *w*^*k*^ and adding bias b_k_ produce the *k*^th^ (FM) *FM*_*ij*_^*k*^ using the tanh function as equation (10).

(10) $$\begin{array}{c} FM_{ij}^{k}=\tanh\left({\left(W^{k}\times x\right)}_{ij}+b_{k}\right). \end{array}$$

By lowering the resolution of FMs, the subsampling layer achieves spatial invariance, in which each pooled FM corresponds to a single FM in the previous layer. Equation (11) is defined as the subsampling function.

(11) $$\begin{array}{c} \alpha_{j}=\tanh\left(\beta \underset{N\times N}{\sum }\alpha_{i}^{n\times n}+b\right). \end{array}$$

where *α*_*i*_^*n*×*n*^ denotes the inputs and *β* and *b*, respectively, denote the trainable scalar and bias. After many convolution and subsampling layers, the final layer is a completely linked structure that carries out the classification process. Each output class has its own neuron. As a result, in the COVID-19 data set, this layer comprises two neurons for each of its classes.

### 2.3. Data set

The database used with the name COVID-X-ray-5k consists of 2084 tutorials and 3100 test images [33]. In this data set, since lateral images are not suitable for identifying the target and according to the radiologist's recommendations, anterior-posterior COVID-19 X-ray images have been used. Radiologists evaluate data set images, and items that do not have exact COVID-19 symptoms are removed. Out of 203 images, 19 images will be deleted, and 184 images with clear signs of COVID-19 will remain. By doing the job in this manner, the community was introduced, as well as a more clearly labeled data set. Of the remaining images, 184 images were used, 100 images were used for network testing, and 84 images were used for network training. Using data augmentation, we increase the number of COVID-19 samples to 420 samples. Due to the small amount of non-COVID pictures in the COVID-chest ray-data set [34], the supplemental ChexPert data set [35] was used. This data set contains 224316 chest X-ray images from 65240 individuals. Totally, 2000 images from the non-COVID-19 data set are used for the training set, and 3000 images are used for the test set.  Table 2 summarizes the total number of photos utilized across all classes (see Table 2 and Figure 3).

Figure 3 illustrates two picture samples from COVID-19 and four standard image samples randomly picked from the COVID-X-ray-5k data set.

### 2.4. Methodology

#### 2.4.1. Presentation of Whales

Two fundamental concepts govern the tuning of deep artificial neural networks: to begin, the structure's parameters must be accurately represented by a FuzzyWOA (candid solution); next, the fitness function must be defined in terms of the problem at hand. The use of FuzzyWOA in DCNN tuning is a distinct phase in the presentation of network parameters. Therefore, to achieve the highest and highest detection accuracy, the essential parameters in DCNN, i.e., weights and FCL, must be clearly defined. In general, FuzzyWOA optimizes the weights and biases used to compute the loss function as the fitness function in the final layer. In other words, whales are used in FuzzyWOA as the last layer's weight and bias values. Three main ways are available for representing the weights and biases of a DCNN as frank solutions of a metaheuristic algorithm: based on vectors, matrices, or binary states [26]. Since FuzzyWOA requires a vector-based model's parameters, this paper uses equation (12) for the candidate solution.

(12) $$\begin{array}{c} \text{Whales}=\left[W_{11}.W_{12}.\;\ldots .W_{nh}.b_{1}.\;\ldots .b_{h}.M_{11}.\;\ldots .M_{hm}\right], \end{array}$$

where *n* denotes the number of input nodes, *W*_*ij*_ denotes the weight of the connection between the *i*_th_ input node and the *j*_th_ hidden neuron, *b*_*j*_ denotes the bias of the *j*_th_ hidden neuron, and *M*_*jo*_ denotes the weight of the connection between the *j*th hidden neuron and the *o*th output neuron. As indicated in Section 2.2, the suggested design is a straightforward LeNet-5 framework. Two structures are utilized in this section: i-6c-2s-12c-2s and i-8c-2s-16c-2s, where C and S denote convolution and subsampling layers, respectively. All convolution layers have a kernel size of 5 × 5, and the scale of subsampling is downsampled by a factor of two.

### 2.5. Loss Function

In designing and proposing the proposed metaheuristic optimizer (DCNN-FuzzyWOA), the task of DCNN training is the responsibility of FuzzyWOA. The purpose of optimization is to obtain the best accuracy, minimizing classification error and network complexity. This target may be calculated using either the whales' loss function or the classification procedure's mean square error (MSE). As a result, the lost function is defined as equation (13).

(13) $$\begin{array}{c} y=\frac{1}{2}\sqrt{\frac{\sum_{i=0}^{N}{\left(o-d\right)}^{2}}{N}}, \end{array}$$

where *o* denotes the computed output, *d* is the desired output, and N denotes the training sample count. Two conditions are defined to terminate FuzzyWOA, including reaching maximum iteration or predefined loss function.

## 3. Results and Discussion

As mentioned in the previous sections, this paper attempts to improve the classic DCNN-FuzzyWOA classifier's accuracy by proposing and designing a fuzzy system to adjust the WOA control parameters. For the DCNN-FuzzyWOA simulation, the population size and maximum iteration are 15. In DCNN, the batch size is 100, and the learning rate is 1. Additionally, the number of epochs examined for each assessment ranges between 1 and 20. The test was conducted in MATLAB-R2020a on a PC equipped with an Intel Core i7-2630QM CPU and 6 GB of RAM running Windows 7, with six distinct runtimes. According to reference [20], the accuracy rate cannot provide sufficient information about the detector's effectiveness.

The suggested classifier's effectiveness in all samples was shown using receiver operating characteristic (ROC) curves. As a result, each sample is assigned an estimated probability of images *P*_*T*_. Following that, a threshold value *T*∈[0.1] was added. Thus, the detection rate was determined for each value. Thus, the obtained values were presented as a receiver operating characteristic (ROC) curve. In general, the concept of ROC diagram curves can be interpreted so that the larger the area under the diagram (AUC), the greater the probability of detection.  Figure 4 shows the result of the ROC curve in the use of DCNN-FuzzyWOA to detect COVID-19. Also, in order to be able to make a fair comparison, a simple DCNN has been used to detect COVID-19. This comparison is made because the test data set, the initial values of the parameters, and the simple CNN structure, i.e., LeNet-5 DCNN, are entirely the same. According to what has been said, the competence and efficiency of DVNN-FuzzyWOA can be considered fair. On the test data set, the ROC curves demonstrate that DCNN-FuzzyWOA beats LeNet-5 DCNN considerably (Figure 4).

The suggested approach was implemented and executed 10 times, with a total training duration of between 4.5 and 11.5 minutes. The proposed classifier (DCNN-FuzzyWOA) for the COVID-19 validation set has a detection power between 99.01% and 100%. Due to the wide range of possible outcomes, the 10 trained DCNN-FuzzyWOA models are ensembled using weighted averaging with validation accuracy as the weights. The DCNN-FuzzyWOA classifier obtains a validation accuracy of 99.27 percent, while the LeNet-5 DCNN classifier achieves a detection accuracy of between 75.08 and 83.98 percent. The resultant ensemble achieves an 86.91 percent detection accuracy on the COVID-19 validation data set. New benchmark models including LeNet-5 DCNN [36], DCNN-GA [20], and DCNN-PSO [37] have been used to prove the efficiency and performance of DCNN-FuzzyWOA in detecting positive and negative cases of COVID-19. The ROC and precision-recall curves for the i-6c-2s-12c-2s and i-8c-2s-16c-2s structures are shown in Figures 5 and 6, respectively. The simulation results show that the DCNN-FuzzyWOA classifier or detector provides better results than other benchmark models.

For a more accurate comparison to understand the power and ability of DCNN-FuzzyWOA to detect positive and negative cases of COVID-19, more than 99.01% of the diagnoses are correct. The false alarm detection rate is less than 0.81%. In general, the trade-off between recall and precision for various threshold levels shows with the precision-recall curve. The greatest area under the precision-recall curve suggests that the accuracy and recall are strong. High precision shows a low false-positive rate, and high-recall indicates a low false-negative rate. Figures 5 and 6 show that DCNN-FuzzyWOA has the largest area under the precision-recall curve. It demonstrates a lower rate of false-positive- and false-negative classifications than other benchmark classifiers (see Tables 3–5).

Tables 3–6 describe the accuracy and computational time findings for the i-6c-2s-12c-2s and i-8c-2s-16c-2s structures. The overall result of the simulation was that the accuracy improved with increasing epoch. For example, in the first epoch, compared to LeNet-5 (77.24), the accuracy increased to 3.84 for DCNN-GA (81.08), 8.63 to DCNN-PSO (89.71), and 1.73 for DCNN-FuzzyWOA (91.44). As shown in Table 3, the improvement in accuracy when 20 epochs are used is 1.57 for DCNN-GA (96.71), 2.05 for DCNN-PSO (98.76), and 1.24 for DCNN-FuzzyWOA (100). The simulation results show that DCNN-FuzzyWOA is more accurate in all epochs. As shown in Tables 4 and 6, processing time in FuzzyWOA is shorter and faster than other methods used.

As the number of epochs rises, the time efficiency of the FuzzyWOA becomes increasingly apparent, as the FuzzyWOA's stochastic structure results in a decrease in the complexity of the search space. It should be noted that the i-8c-2s-16c-2s structure findings in Tables 5 and 6 corroborate the previous conclusion about the i-8c-2s-16c-2s network. As a result, FuzzyWOA can significantly increase the performance of DCNNs with i-8c-2s-16c-2s and i-6c-2s-12c-2s structures. Data science experts believe that the best results can be shown using overall accuracy, ROC curve, F1-Score. Therefore, Table 7 examines the F1-Score in structures i-2s-6c-2s-12c and i-2s-8c-2s-16c.

As shown in Table 7, the results obtained from FuzzyWOA are more appropriate and encouraging than the other methods used. So that, in the twentieth epoch, in the structure of i-2s-6c-2s-12c, the value of F1-Score reaches 100%.

## 4. Conclusion

In this paper, using AI tools, i.e., a combination of DCNN, WOA, and fuzzy logic, an accurate model is designed and proposed to detect the positive and negative cases of COVID-19 using X-ray. In addition to using the COVID-Xray-5k benchmark data set, the DCNN-PSO, DCNN-GA, and DCNN classic models were used for a fair comparison of the proposed detector or classifier. Analysis of simulation results provided comparable and significant results for the proposed DCNN-FuzzyWOA model. Experts also confirmed the relationship between the results and clinical results. One of the most significant reasons for the optimal performance of the DCNN-FuzzyWOA model is the adjustment of WOA control parameters by the fuzzy system and the determination of a clear boundary between the exploration and extraction phases in the search space of the WOA trainer algorithm. All training algorithms used to train the two convolutional networks were compared in terms of accuracy, processing time, F1-Score, and curves of ROC and precision-recall. The results showed that FuzzyWOA had a more encouraging performance than the other methods used. In terms of structure, the i-2s-6c-2s-12c architecture has been more successful. Of course, despite getting good results from DCNN-FuzzyWOA, larger data sets than COVID-19 are needed to achieve higher accuracy with more excellent reliability.

## Figures and Tables

**Figure 1:** A proposed fuzzy model for setting parameters $\overset{⟶}{\alpha }$ and $\overset{⟶}{C}$.

**Figure 2:** The LeNet-5 DCNN's architecture.

**Figure 3:** Images random from the COVID-X-ray-5k data set [33].

**Figure 4:** ROC curves for DCNN-FuzzyWOA and LeNet-5.

**Figure 5:** Curves of ROC and precision-recall for the i-6c-2s-12c-2s models.

**Figure 6:** Curves of ROC and precision-recall for the i-8c-2s-16c-2s models.

**Table 1:** Applied fuzzy rules.

If (NFV is low) and ($\overset{⟶}{\alpha }$ is low), then (Δ*α* is ZE)
If (NFV is low) and ($\overset{⟶}{\alpha }$ is medium), then (Δ*α* is NE)
If (NFV is low) and ($\overset{⟶}{\alpha }$ is high), then (Δ*α* is NE)
If (NFV is medium) and ($\overset{⟶}{\alpha }$ is low), then (Δ*α* is PO)
If (NFV is medium) and ($\overset{⟶}{\alpha }$ is medium), then (Δ*α* is ZE)
If (NFV is medium) and ($\overset{⟶}{\alpha }$ is high), then (Δ*α* is NE)
If (NFV is high) and ($\overset{⟶}{\alpha }$ is low), then (Δ*α* is PO)
If (NFV is high) and ($\overset{⟶}{\alpha }$ is medium), then (Δ*α* is ZE)
If (NFV is high) and ($\overset{⟶}{\alpha }$ is high), then (Δ*α* is NE)
If (NFV is low) and ($\overset{⟶}{C}$ is low), then (Δ*C* is PO)
If (NFV is low) and ($\overset{⟶}{C}$ is medium), then (Δ*C* is PO)
If (NFV is low) and ($\overset{⟶}{C}$ is high), then (Δ*C* is ZE)
If (NFV is medium) and ($\overset{⟶}{C}$ is low), then (Δ*C* is PO)
If (NFV is medium) and ($\overset{⟶}{C}$ is medium), then (Δ*C* is ZE)
If (NFV is medium) and ($\overset{⟶}{C}$ is high), then (Δ*C* is NE)
If (NFV is high) and ($\overset{⟶}{C}$ is low), then (Δ*C* is PO)
If (NFV is high) and ($\overset{⟶}{C}$ is medium), then (Δ*C* is ZE)
If (NFV is high) and ($\overset{⟶}{C}$ is high), then (Δ*C* is NE)

**Table 2:** The COVID data set's image categories [33].

Category	COVID-19	Normal
Training set	84 (420 after augmentation)	2000
Test set	100	3000

**Table 3:** Accuracy and STD for the i-2s-6c-2s-12c structure.

Epoch	DCNN-FuzzyWOA		DCNN-PSO		DCNN-GA		LeNet-5	
	Accuracy	STD	Accuracy	STD	Accuracy	STD	Accuracy	STD
1	91.44	N/A	89.71	0.48	81.08	0.11	77.24	0.71
2	91.94	N/A	90.08	0.22	82.05	0.24	78.41	0.23
3	92.09	N/A	90.89	0.45	83.40	0.13	78.99	0.41
4	92.73	N/A	91.53	0.43	85.66	0.12	79.66	0.95
5	93.51	N/A	92.66	0.34	86.91	0.35	80.11	0.19
6	93.84	N/A	92.99	0.38	87.25	0.16	81.25	0.33
7	94.11	N/A	93.35	0.37	88.82	0.24	82.32	0.71
8	94.62	N/A	93.83	0.24	89.33	0.18	83.41	0.91
9	94.77	N/A	94.16	0.33	90.14	0.16	84.53	0.15
10	95.14	N/A	94.51	0.32	90.57	0.42	85.82	0.36
11	95.87	N/A	94.93	0.31	91.27	0.16	86.28	0.37
12	96.29	N/A	95.10	0.30	91.89	0.30	87.23	0.26
13	96.71	N/A	95.65	0.29	92.51	0.21	89.51	0.83
14	96.64	N/A	96.27	0.44	93.34	0.39	90.19	0.31
15	97.88	N/A	96.69	0.23	93.97	0.17	91.50	0.66
16	98.07	N/A	97.04	0.22	94.43	0.41	92.08	0.47
17	98.60	N/A	97.80	0.19	94.82	0.26	93.61	0.62
18	99.13	N/A	98.13	0.67	95.60	0.18	94.33	0.59
19	99.72	N/A	98.61	0.12	96.52	0.33	94.91	0.51
20	100	N/A	98.76	0.09	96.71	0.10	95.14	0.13

**Table 4:** Time required to compute and standard deviation for the i-2s-6c-2s-12c structure.

Epoch	DCNN-FuzzyWOA		DCNN-PSO		DCNN-GA		LeNet-5	
	Time	STD	Time	STD	Time	STD	Time	STD
1	85.91	N/A	108.55	1.04	115.01	0.78	127.08	0.81
2	115.87	N/A	199.43	1.02	161.76	1.71	195.20	1.07
3	184.65	N/A	283.71	2.08	221.95	2.41	238.85	2.58
4	222.41	N/A	305.86	1.07	260.74	1.09	299.50	1.17
5	291.33	N/A	390.29	1.23	317.55	4.99	310.17	4.37
6	301.96	N/A	448.91	2.11	361.34	3.14	422.39	1.08
7	345.17	N/A	519.57	1.56	433.98	2.08	531.81	2.09
8	379.86	N/A	589.39	1.84	549.27	1.19	579.27	4.01
9	405.16	N/A	618.28	2.42	625.10	1.78	536.90	1.28
10	476.22	N/A	697.68	3.86	677.31	2.77	640.33	4.65
11	495.57	N/A	737.70	3.07	731.79	1.18	678.88	2.65
12	511.79	N/A	793.32	1.73	792.03	3.34	723.74	1.59
13	577.73	N/A	836.15	1.66	841.50	4.28	791.83	2.66
14	601.63	N/A	889.04	2.37	881.53	3.11	845.70	2.13
15	647.85	N/A	923.17	2.09	903.72	1.56	936.62	1.83
16	690.33	N/A	978.64	1.88	930.18	4.66	1005.78	3.11
17	728.36	N/A	1001.79	3.77	982.04	1.23	1075.29	2.64
18	774.14	N/A	1060.8	1.91	1030.77	1.11	1103.21	2.23
19	834.71	N/A	1101.08	2.14	1161.20	3.28	1152.56	3.01
20	880.44	N/A	1186.61	1.89	1240.11	4.79	1256.07	1.74

**Table 5:** Accuracy and STD for the i-2s-8c-2s-16c structure.

Epoch	DCNN-FuzzyWOA		DCNN-PSO		DCNN-GA		LeNet-5	
	Accuracy	STD	Accuracy	STD	Accuracy	STD	Accuracy	STD
1	90.23	N/A	87.09	0.20	80.38	0.19	76.33	1.05
2	90.89	N/A	88.40	0.19	80.79	0.17	77.00	0.89
3	91.63	N/A	88.87	0.11	81.15	0.26	78.09	2.32
4	91.81	N/A	90.25	0.14	81.68	0.31	79.34	3.76
5	92.33	N/A	90.66	0.27	82.34	0.19	80.55	1.90
6	93.26	N/A	91.23	0.23	83.71	0.14	81.21	4.58
7	93.19	N/A	92.00	0.30	84.53	0.21	82.38	3.72
8	93.99	N/A	92.19	0.18	85.61	0.16	82.79	1.18
9	94.20	N/A	92.85	0.19	86.67	0.28	83.48	0.52
10	94.18	N/A	93.34	0.36	87.41	0.15	84.31	2.63
11	95.51	N/A	93.28	0.15	88.52	0.22	85.63	2.88
12	95.79	N/A	94.47	0.09	89.05	0.16	86.84	5.23
13	96.37	N/A	95.69	0.11	89.98	0.14	87.37	4.19
14	97.31	N/A	95.91	0.22	90.37	0.32	89.06	3.55
15	97.72	N/A	96.38	0.06	91.25	0.28	90.71	5.10
16	97.92	N/A	96.74	0.33	92.40	0.13	91.76	1.74
17	98.30	N/A	97.29	0.31	93.71	0.19	92.25	3.19
18	98.65	N/A	97.84	0.08	94.64	0.25	93.16	1.53
19	99.08	N/A	98.07	0.28	95.18	0.18	94.72	0.68
20	99.55	N/A	98.63	0.12	96.31	0.12	95.08	4.80

**Table 6:** Time required to compute and standard deviation for the the i-2s-8c-2s-16c structure.

Epoch	DCNN-FuzzyWOA		DCNN-PSO		DCNN-GA		LeNet-5	
	Time	STD	Time	STD	Time	STD	Time	STD
1	83.35	N/A	110.21	1.04	117.43	1.53	154.51	3.74
2	118.24	N/A	200.17	1.02	158.53	1.64	202.19	2.83
3	165.75	N/A	275.68	2.08	215.37	2.57	244.28	1.97
4	218.60	N/A	311.72	1.07	262.71	1.67	315.37	2.55
5	293.19	N/A	364.33	1.23	321.14	0.91	376.63	3.77
6	321.71	N/A	446.17	2.11	365.31	3.16	418.18	1.84
7	353.63	N/A	528.91	1.56	442.28	2.27	546.92	3.74
8	384.28	N/A	593.53	1.84	550.28	2.16	573.11	4.58
9	410.46	N/A	625.34	2.42	628.31	1.13	535.63	2.63
10	496.39	N/A	670.81	3.86	680.32	4.28	632.27	0.63
11	508.77	N/A	741.73	3.07	734.62	5.33	689.81	3.27
12	542.91	N/A	799.84	1.73	783.49	2.59	722.35	3.36
13	596.72	N/A	842.59	1.69	853.78	1.49	793.44	1.25
14	663.85	N/A	891.70	2.37	892.75	2.27	835.23	2.80
15	689.51	N/A	928.91	2.08	913.36	1.56	947.95	2.33
16	734.38	N/A	974.32	1.87	936.77	2.23	1025.52	4.20
17	770.41	N/A	1011.30	3.76	980.19	1.44	1098.37	0.76
18	829.13	N/A	1063.85	1.95	1032.83	1.78	1110.50	1.58
19	857.67	N/A	1127.63	2.32	1163.27	2.56	1153.48	0.99
20	945.61	N/A	1201.21	1.89	1262.46	5.11	1398.13	1.81

**Table 7:** Comparison of F1-Score in structures i-2s-6c-2s-12c and i-2s-8c-2s-16c.

Structure	i-2s-6c-2s-12c				i-2s-8c-2s-16c			
	F1−score %				F1−score %			
Epoch	DCNN-FuzzyWOA	DCNN-PSO	DCNN-GA	LeNet-5	DCNN-FuzzyWOA	DCNN-PSO	DCNN-GA	LeNet-5
1	89.10	89.71	73.21	70.06	89.89	80.51	77.84	0.10
2	89.13	87.86	73.87	78.41	90.25	81.19	78.45	0.42
3	89.89	89.04	75.62	73.24	90.63	82.27	79.86	1.53
4	90.78	90.18	75.75	74.93	91.03	83.97	81.68	2.46
5	91.20	92.14	77.19	75.08	91.19	84.23	83.54	1.90
6	91.22	92.31	77.73	75.62	91.43	84.35	84.94	2.68
7	91.49	92.45	78.62	76.80	93.19	92.00	85.53	1.52
8	91.98	92.45	79.79	76.71	92.44	86.54	86.54	1.18
9	93.44	92.83	80.81	79.82	94.08	86.11	87.68	0.52
10	93.47	93.10	82.11	80.74	94.02	88.37	87.41	1.27
11	94.19	93.13	85.51	80.97	94.51	88.62	88.52	1.36
12	94.28	93.27	91.89	83.44	95.79	89.49	89.18	1.89
13	95.31	93.76	88.48	87.32	96.37	90.13	89.57	2.25
14	95.77	95.00	93.35	88.18	97.31	91.91	89.96	1.46
15	97.01	95.13	89.22	89.04	95.11	92.81	90.14	3.91
16	97.47	95.50	90.67	89.49	95.34	92.65	90.72	1.23
17	97.90	95.89	91.34	89.78	95.89	94.29	93.71	2.85
18	98.53	96.31	91.52	90.08	96.51	95.81	94.64	0.79
19	98.99	96.66	96.25	91.37	97.00	96.07	94.89	0.91
20	100	96.97	93.15	91.45	97.31	96.73	94.32	2.89

## Data Availability

Data are available and can be provided over the emails querying directly to the author at the corresponding author (abbas.saffari@birjand.ac.ir).
